RETRACTED

# Early Detection of Autism Spectrum Disorders (ASD) with the Help of Data Mining Tools

**DOI:** 10.1155/2022/1201129

**Published:** 2022-05-23

**Authors:** Ammar Akram Abdulrazzaq, Sana Sulaiman Hamid, Asaad T. Al-Douri, A. A. Hamad Mohamad, Abdelrahman Mohamed Ibrahim

**Affiliations:** ^1^Department of Medical Laboratory Techniques, Al-Maarif University College, Al-Anbar, Iraq; ^2^Al-Farahidi University, Communication Technical Engineering, Baghdad, Iraq; ^3^Department of Dental Industry, College of Medical Technology, Al-Kitab University, Iraq; ^4^Department of Medical Laboratory Techniques, Dijlah University College, Baghdad 10021, Iraq; ^5^The University of Mashreq, Research Center, Baghdad, Iraq; ^6^Accounting and Financial Management, School of Management Studies, University of Khartoum, Sudan

## Abstract

Autism is a disorder of neurobiological origin that originates a different course in the development of verbal and nonverbal communication, social interactions, the flexibility of behavior, and interests. The results obtained offer relevant information to reflect on the practices currently used in assessing the development of children and the detection of ASD and suggest the need to strengthen the training of health professionals in aspects such as psychology and developmental disorders. This study, based on genuine and current facts, used data from 292 children with an autism spectrum disorder. The input dataset has 20 characteristics, and the output dataset has one attribute. The output property indicates whether or not a certain person has autism. The research study first and foremost performed data pretreatment activities such as filling in missing data gaps in the data collection, digitizing categorical data, and normalizing. The features were then clustered using *k*-means and *x*-means clustering methods, then artificial neural networks and a linguistic strong neurofuzzy classifier were used to classify them. The outcomes of each strategy were examined, and their respective performances were compared.

## 1. Introduction

Autism spectrum disorders (ASD) are a collection of illnesses characterized by anomalies in the formation and function of neural circuits. Recent epidemiological studies suggest an increase in autism cases [1], for example, 5 cases per 10,000 in 1985, but now 1 case per 100 children and adolescents. It is unknown if this is related to a change in diagnostic criteria or an actual rise in occurrence. It is probable because other illnesses that influence language, learning, and/or mental retardation are now classified better. The sex ratio is 4 to 11. Despite the lack of consensus, it appears that the peak occurrence age is 8 years; mental retardation: 75% (45-60% in other studies) [2]. These percentages are more akin to typical autism, with PDD being less common and AS being almost nonexistent, with roughly 30% of cases associated with mental retardation. These people are probable carriers of unknown illnesses in which autism is one aspect of a more complex neurological picture. Secondary autisms, on the other hand, occur when another pathology is found in the same person with ASD, usually a rare disease that has been linked to autism—fragile X syndrome, tuberous sclerosis, Angelman syndrome, rubella, etc.—or where it is suspected that all manifestations are part of the same syndromic complex, severe intellectual disability (PID), cognitive disability (CD), ataxia (motor difficulties), blindness and other eye ailments (BAE), deafness (BAE), hyperactivity (hyperactivity), anxiety (anxiety), and insomnia (insomnia) [3]. There is a lot of discussion in the literature and several research about the early detection of ASD [4]. Most studies in this field agree that early intervention can help these people overcome their shortcomings (IQ, social skills, coping skills, etc.) and help them integrate. The consensus is that these improvements do not suggest a cure but rather a reduction in family and social load and patient well-being. For these reasons, many studies have concentrated on finding instruments that allow early identification, both in high-risk groups like autistic siblings and in general or low-risk populations, the Autism Observation Scale for Infants (AOSI) for studies of autistic siblings and the Childhood Autism Spectrum Test (CAST) for children aged 4 to 6. The Autonomous Scale has been validated in Arabic nations [5].

RETRACTED

Data mining is a search for knowledge. Data mining seeks out previously unknown patterns. In other terms, data mining is a set of technologies that allow the creation of meaningful expressions from raw and unintelligible data. When the objective of data mining is considered, it is similar to ore mining [6].

Technology is heavily employed in medicine as in every field. With the advancement of technology, new medical equipment and treatment procedures are being produced. These methods, which are constantly evolving in hardware and software, allow for more professional diagnosis and treatment [7]. Because medicine deals with human health, it is critical to encourage and support R&D. Many treatments rely on early diagnosis. Delaying treatment may cause disease progression and make treatment more difficult. It can potentially result in irreversible losses. For these reasons, data mining strategies to help doctors diagnose and treat patients are common in the literature [8]. Medicine's technological studies are a mix of numerous fields. Because vital information from the patient or examination findings cannot be reviewed without one or more physicians who are experts in the condition and diagnosis, nonexperts in the subject cannot evaluate disease-related findings. To assess if a person has an illness, a specialist must know precise details about the disease. Otherwise, erroneous diagnoses and treatment delays may occur. This may cause more serious issues. As a result, professionals in the subject must be consulted when applying information technologies in diagnosis. Experts agree that collecting the parameters and analyzing them later is best. These analyses require someone who can use information technologies to translate expert data into relevant information.

RETRACTED

As a result, the collaboration between disciplines is critical to a successful study. There are classification procedures employing logistic regression, naive Bayes, artificial neural networks, and linguistic strong neurofuzzy classifiers and any classification. No method of clustering was found. This study used data pretreatment approaches such as filling in missing data and standardization, followed by a clustering method that was lacking in the literature and two unproven methods for classification. The study compares the methodologies' success rates using criteria including accuracy, sensitivity, determination, and *F*-measure to add to the literature. Artificial neural networks and strong linguistic neurofuzzy classifier approaches were employed for classification. Regarding estimation accuracy, classification methods outperform clustering methods in data on autism spectrum disorder in children. The linguistic strong neurofuzzy classifier approach has a greater success rate than many other methods in the literature, properly classifying all data.

## 2. Methodology

### 2.1. Classification Method

#### 2.1.1. Artificial Neural Networks

Artificial neural networks (ANNs) are an algorithm inspired by how the human brain works. Biological findings of neurophysiologists and psychologists on how neural networks work are used as its basis. These biological findings were systematized structurally and functionally, and a mathematical model was tried to be created. This model is called the neural network model [9].

#### 2.1.2. Linguistic Strong Neurofuzzy Classifier

The linguistic strong neurofuzzy classifier (DKSBS) classifies data. Before classifying, determine the relevance of the features. Fuzzy inference is used to rank the features' relevance [10]. Thus, high-importance features are selected while low-importance features are disabled. This is the key distinction between classical and fuzzy logic. Sets can be made up of elements in fuzzy logic. In other words, the state of being an element with one and not being an element with 0 can be represented as 0.3 and 0.5 degrees. Also, since elements do not have to be in the same cluster, an element can be included in one cluster at 0.3 and another at 0.5. This eliminates the clear separation between black and white in classical clusters, allowing for grey spaces. So, by using a fuzzy technique, partial memberships can be established. To classify the features, the fuzzy inference is utilized first. The success rate of training the ANN is high due to the inclusion of fuzzy inference features. Memory is saved by not using attributes that do not split sets. This condition not only speeds up the process but also reduces costs. There is no need to use certain features if the classification success does not diminish when they are removed [8], because in real-life problems, the influence degree of the solutions developed can be different. The goal is to find faster and more accurate solutions. In this sense, the linguistically powerful fuzzy neuroclassifier provides a solution very near to real-life challenges. The data mining process is divided into two steps. First, the preprocessing stage of identifying the importance of the features is carried out. The artificial neural network is then trained using these importance levels and performed classification. The linguistic strong neurofuzzy classifier distinguishes itself from other classification methods by performing feature detection using fuzzy inference. The linguistic strong neurofuzzy classifier employs fuzzy rules to classify features. Fuzzy rules gradually define the features. Blurring frees the system from binary replies like yes or no. In other words, rather than being categorical, whether an attribute affects the outcome is described as “few,” “there is,” or “a lot.” So, fuzzy inferences become more human-like.

RETRACTED

### 2.2. Clustering Method

#### 2.2.1. *K*-Means

Clustering is the process of grouping components together. Clustering is a popular strategy for grouping datasets and disclosing crucial and secret information [11]. The distinction between clustering and classification, another data mining process, is that classes in clustering are not predetermined. *K*-means is one of the oldest nonhierarchical clustering algorithms. Clustering uses unsupervised learning. In other words, clustering is not preset. Clusters are constructed by establishing the cluster's center points. The parameter *k* specifies the number of clusters. Because the *K* parameter also contains the number of cluster centers, it must be entered before employing the *K*-means algorithm. When determining clusters, the goal is to have the most in-group and least intergroup similarities. Distances between data points are used while forming similar clusters. Here, the appropriate number of cluster centres is determined (*k* parameter), and the distances of each element to these cluster centers are calculated one by one. Due to noncomputation, each data is included in the nearest cluster cen. The new cluster centres are recalculated, as are the distances between each element and the new cluster centres. This cycle repeats until the set with no element changes. To finish the procedure, each element is assigned to the cluster in which it was found last. The elements that share the most similarities are grouped following the algorithm's distance calculations. The main flaw of *k*-means is that it cannot predict how many clusters the data will be divided into. If the number of clusters in the data is known, the *k* parameter can be entered, or the most relevant one can be identified by inputting different *k* parameters.

#### 2.2.2. *X*-Means

*K*-means is a well-known clustering technique. The popularity of *K*-means is due to its simple structure and high model performance rate. However, despite its popularity, it has certain flaws. The user must supply a fixed value for the *k* parameter, representing the number of clusters. Limiting the number of clusters to a set *k*-value means ignoring other options. *X*-means stores the data in a *kd*-tree and stores the statistics for each stage. The statistical data also contains a list of centers to consider for a certain region. So, by comparing all options, the best one can be chosen. Pelleg and Moore developed the *X*-means method in 2000 as an upgraded version of the *K*-means algorithm. It was built to fill in the gaps in the *K*-means algorithm and to use the *K*-means algorithm's working style [12].

The method cannot calculate the number of clusters, which is viewed as a shortcoming of *X*-means and *K*-means. Instead of a predetermined number of clusters, *X*-means specifies an appropriate range. *X*-means may estimate the number of clusters it considers optimal from this range of values. The *X*-means structure runs the *K*-means algorithm progressively. Each time *K*-means creates subsets, it decides which centres to divide them between. Calculate the Bayes information criteria to make division judgments. These are the best results of existing centres (parent) and newly developed offspring (child). The *k* parameter values used to score the model selection criteria are kept adjacent to the cluster centres. So, the centre positions can be studied attentively. The procedure starts with *k* equal to the range's lower limit and adds new centres until the upper limit is reached. During these operations, the best-scoring centroid set is noted. The new score is added if the following transaction's score is higher than the system's score. So, the list is always updated. A list of probable centroids for locations within a region is kept recursively updated. Its job is to update the region's centre points with the proper values. It starts by recording the randomly generated centre points equal to the *k* parameter list's smallest integer. The new values are updated as better ones are found. Finally, the highest-valued centres are outputs.

RETRACTED

### 2.3. Preprocessing Techniques

Data mining methods may collect incomplete data. In such circumstances, missing data analyses are possible. At the same time, it is preferable to repair missing data to increase the dataset's quality. Analysing entire data also helps improve the method's success rate [13]. Missing data correction is part of preprocessing. It is possible to correct missing data by removing records or completing them in various ways. There are numerous approaches for completing missing data in the literature. A value assigned by taking into account the features of other data (such as mean, mode, or median) or values determined as a consequence of guesses might be used to fill in the missing values (regression analysis, hot deck value with Naive Bayes assignment, decision trees, expectation-maximization, and multiple assignment). This study assigned values based on other data's properties to fill in the gaps. The dataset's frequency was evaluated, and the value with the highest frequency was utilized to fill in the gaps.

Data mining is commonly used nowadays to extract meaning from data. Data mining is the process of discovering knowledge through data collecting, preprocessing, transformation, applying data mining tools, and assessing the results. The quality of the data acquired is important in enhancing the method's success rate. Many data preparation techniques exist to increase data quality. Preprocessing approaches include filling in missing data, eliminating noisy data, assessing feature relevance, and normalising particular features. Preprocessing methods and normalisation were employed to fill in missing data. The literature accepts various types of normalisation. Normalization methods include *Z*-score, min-max, median, and Sigmoid. Several normalising approaches can be employed concurrently. This study employed min-max normalisation.

## 3. Application

### 3.1. Autism Spectrum Disorder Dataset

This study used a subset of genuine ASD data for youngsters. The dataset used is called Autism Spectrum Disorder Screening Data for Children [14]. The dataset was developed using the latest parameters acknowledged in the literature for ASD diagnosis. The ASD Tests app gathered the answers. The application has age-specific categories. Each category has ten questions, each illustration to help users choose the correct answer. Participants were told their data would be kept confidential and used only for research. Participants were briefed on the research's goal, privacy policy, and data use before completing the evaluation. The data collection includes ten items measuring autism spectrum disorder and demographic data. This test included data from three subgroups, totalling 1100 persons. Youth and adults make up the groups. ASD diagnoses are divided into groups based on the questions addressed. The produced dataset for children contains 292 samples, and only this subset was used in this investigation. Data kinds include numerical and categorical. Some data samples in the collection are missing. 20 attributes were used as inputs because they contained information on individuals' general and health state, and 1 attribute was used as output since it included the individual's autistic status. The attribute field “kind of screening method” expresses the individual's age range. In other words, it shows which child, teen, or adult group the autism screening tester belongs to. Only the kid subset was employed in this investigation. Data was unnecessary as it was all about the kids. So, it was eliminated from the dataset. So, there are now only 19 input parameters.  Table 1 details the qualities and questions.

RETRACTED

The attribute “kind of screening procedure,” which indicates which age category the dataset applies to, has been removed from the dataset. The autism status of the Boolean individual was employed as a class label. First, all features were translated into numerical values in the study. Data pretreatment techniques such as filling in missing data and standardising data between 0 and 1 were performed to evaluate the dataset more efficiently. The data were then categorised with DKSBS and grouped with *k*-means and *x*-means. The number of neurons employed in the planned feedforward ANN on the success rate was investigated. The data were divided into 70% training and 30% testing to examine the model success rate of classification approaches. When the data were categorized by artificial neural networks and DKSBS, the success rate was 100% in the test and training sets. Clustering algorithms lack a pretutorial. Thus, the clustered data were used for both training and testing. 89.73% success rate in *k*-means and 88.0% success rate in *x*-means.

RETRACTED

### 3.2. Findings and Evaluation

Many studies on autism use data mining approaches, according to the literature. Vellanki et al. [15] addressed this issue in his work, stating that the data was outdated, despite the positive results. So, he stressed the need to work with current data. Aloumi et al. [16] supplied the current scale data with a fresh investigation. Aloumi et al. [16] used a subset of data from scientific articles for children in this investigation. The dataset used 292 samples and 21 characteristics. Because the data are relatively new, the findings of this study were compared to other investigations.

The dataset originally had numeric and textual expression variables. The methods employed for normalization and classification cannot be used with string expressions. So, first, the dataset was converted to numerical values. This conversion converts category data tagged with string expressions to numeric expressions. For example, gender categorical data has been replaced by 0 and 1. Ethnicity and residency are also designated consecutively starting at 1.

After digitizing the data, the frequency of each characteristic was recovered. The dataset's null values are filled with the most frequent value. Then, the values acquired with the min-max normalization approach, which has the best success rate of all normalizing methods, were constructed. Part of the dataset is allocated for training and a half for testing to compare the methods' success. The literature shows that several ratios are employed, but 70% of training data and 30% of test data are most typical. This study used 205 randomly selected training samples (70%) and 87 randomly selected testing samples (30%) to comply with the general methodology. Data were grouped using *K*-means and *X*-means.

#### 3.2.1. Results Obtained with Artificial Neural Network

With the designed feedforward ANN, the effect of the number of neurons used on the success rate was examined, and models with different structures were tested. The performance of ANN is given in Figure 1.

When the success rate of the designed models is examined, it has been seen that a very high rate of success has been achieved. Among the models designed with different neuron numbers, the highest performance was seen in the model designed using 20 neurons in the input layer, 5 neurons in the two hidden layers, and 2 neurons in the output layer. Success was achieved with an accuracy of 100% in the training set and 98.85% in the test set. All samples in the training set are classified correctly, while only one sample in the test dataset is classified incorrectly. As seen in Figure 1, increasing the number of neurons in the hidden layer is not directly proportional to the increase in the success rate. While increasing the number of neurons increases the model's success rate for some datasets, it decreases the model's success rate for some datasets. Therefore, instead of always adopting a fixed approach related to using too many or too little of the number of neurons, choosing the most successful model by determining several alternatives can increase the success rate. The ANN model with the highest success rate is shown in Figure 2.

RETRACTED

The ROC curve (receiver-operating characteristic) drawn for the test data of the trained network is given in Figure 3.

As seen in Figure 3, the area under the ROC curve (AUC) value is very close to 1. This shows that a very high success was achieved in the classification made on the test data. The error matrix drawn for the test data of the trained network is given in Figure 4.

As shown in Figure 4, a very high part of the classification performed by the trained network for the test dataset was predicted correctly, and only one sample was misclassified. This means a very high success for the test data. When the error values produced by the network for the test data are examined in detail, the MSE value is 4.822*e*-04; it is seen that the RMSE value is 0.022. As can be seen from the MSE and RMSE values for the training data of the trained network, the error values of the network are quite low. The accuracy, sensitivity, determination, and *F*-measure values of the trained network for the test data are 0.989, 0.974, 1, and 0.987, respectively. This shows that the trained network gives very successful results in the test data.

#### 3.2.2. Results Obtained with the Linguistic Strong Neurofuzzy Classifier

Firstly, feature selection was performed with DKSBS, and then, classification was performed. The data was divided into 70% training and 30% test data in the classification. When the classification results were examined, it was seen that 100% success was achieved in the training and test data. When the error values calculated for the training data of the method are examined, it is seen that the MSE value is 3.099*e*-32, and the RMSE value is 1.760*e*-16. The feature selection performed was determined by looking at the importance level of the features. The importance levels of the features are determined by DKSBS. The order of the numbered features are the same as the order in Table 1 and progressed sequentially from 1 to 19. Considering the importance levels determined by the linguistic strong neurofuzzy classifier on the features for classification, it is seen that groups with five different importance levels are formed. If these groups are to be rated from 5 to 1, with 5 of them being the most important, attributes with 5 significance levels 1, 2, 3, 5, 6, 7, 10, 18, and 4 importance attributes with 4 and 3 significance levels 8, 9, 11, 12, 13, 14, and 15. The numbered ones are the attribute number 16 with a significance level of 2 and the attribute number 17 with a severity level of 1. The significance level of attribute number 19 is set to 0—the contribution degrees of the features expressed by the linguistic strong neurofuzzy classifier. The child is with attributes 1, 2, 3, 5, 6, 7, and 10 in Table 1, whether he usually notices small sounds when others are not hearing it, whether he usually focuses on the whole picture rather than the small details, whether he can easily follow the conversation of several different people in a social group, whether he knows how to continue the conversation with the candidates, and whether he is good at social conversation, when he reads a story; the character and the features that have the most impact on the classification were determined whether they had difficulty in deciphering their intentions or feelings and whether they found it difficult to make new friends. The final score was obtained based on the screening method's scoring algorithm. Expressed with the number 4 as the second most effective attribute, he found it easy to go back and forth between different activities. The third most effective attributes are expressed with the numbers 8, 9, 11, 12, 13, 14, and 15, whether he likes to play with other children when he is in preschool education and whether he can easily understand what someone is thinking or feeling, just by looking at their face, the age of the individual in years, the information of whether the individual is male or female, the information of the individual's ethnic origin, and the information of the individual's jaundice. It is the information of whether to be born with or not and whether any individual family member has PDD. The fourth most effective attribute is expressed with the number 16, information of the country in which the individual resides. The fifth most effective attribute is expressed with the number 17; it is the information whether the user has used a scanning application before or not. The training performance of the linguistic strong neurofuzzy classifier is shown in Figure 5.

RETRACTED

As shown in Figure 5, the error values of the linguistically strong neurofuzzy classifier are quite low. The error matrix drawn for the test data after the linguistic strong neurofuzzy classifier is trained is given in Figure 6.

As shown in Figure 6, the classification performed by the trained linguistic strong neurofuzzy classifier for the test dataset is all correct. The test data's accuracy, sensitivity, determination, and *F*-measure values performed by the trained linguistic strong neurofuzzy classifier are 1, 1, 1, and 1, respectively. This shows that all of the training data are classified correctly.

#### 3.2.3. Results with *K*-Means

Clustering algorithms are methods without prior tutorials, and the data classes are not predetermined. For this reason, parents were not separated as training and test data; all of them were used for training. In the *k*-means algorithm, the number of clusters expressed by the *k* parameter should be determined beforehand and given to the algorithm before running. There are two classes of data in this study to show whether it is OSB or not. Therefore, two clusters were desired when creating the clusters, so the *k* parameter was entered as two, and the data were clustered into two. When the classes of the data clustered with the *K*-means algorithm are compared with the real cluster classes, 262 of the 292 data in total were correctly classified, and the accuracy of the classification was 89.73%. The real classes and the classes were obtained with *K*-means.

As seen in Figure 7, the classes of the data clustered with the *K*-means algorithm were mostly predicted correctly, and the total number of incorrectly predicted samples was 30. Accuracy, sensitivity, determination, and *F*-measure values of the data clustered with the *K*-means algorithm are 0.897, 0.821, 0.979, and 0.892, respectively.

#### 3.2.4. Results with *X*-Means

The *X*-means algorithm is a more up-to-date clustering method created by the development of the *K*-means algorithm. *X*-means is an improved version of *K*-means besides using the working structure of *K*-means. It works by specifying a range instead of determining the number of clusters as a fixed value. Thus, the algorithm determines the most suitable number of clusters for the dataset. While determining the number of clusters, the Bayesian information criterion is used to determine the best number of clusters. In this study, the number of clusters in the *X*-means algorithm, which was run by entering the class range between 2 and 4, was determined as 2 by the algorithm. When the classes of data clustered in two with the *X*-means algorithm were compared with the real cluster classes, 257 out of 292 data were correctly classified, and the classification accuracy was 88.02%. The real classes and the classes were obtained with *X*-means. The error matrix drawn for the results obtained with the *X*-means algorithm is given in Figure 8.

As seen in Figure 8, the data classes clustered with the *X*-means algorithm were mostly predicted correctly, and the total number of incorrectly predicted samples was 35. Accuracy, sensitivity, determination, and *F*-measure values of the data clustered with the *X*-means algorithm are 0.880, 0.781, 0.986, and 0.871, respectively.

RETRACTED

#### 3.2.5. Comparison of the Prediction Achievements of Autism Spectrum Disorder Data for Children Analyzed with Different Methods

In this study, the subset of the ASD dataset for children was classified with ANN and DKSBS and clustered with *K*-means and *X*-means methods. The performance values of the methods used are given in Figure 9.

As seen in Table 1, although the classification success rate with ANN is quite high, the highest success rate was obtained with DKSBS. In the classification made with DKSBS, 100% accuracy was achieved for training and test data. This means that the linguistic strong neurofuzzy classifier correctly classifies all samples in the dataset. When the success rates of clustering methods are examined, it is seen that they are less successful than classification methods in general, and the results obtained with the *K*-means method are more successful than the *X*-means method. The accuracy, sensitivity, determination, and *F*-measure values for the training datasets of the methods used are given in Figure 10.

Figure 10 shows the accuracy, sensitivity, determination, and *F*-measure values calculated for the training data of the classification and clustering methods. As can be seen, all values calculated in the classification methods are 1. In clustering methods, on average, the calculated values for *K*-means are higher than *X*-means. The accuracy, sensitivity, determination, and *F*-measure values for the test datasets of the methods used are given in Figure 11.

As seen in Figure 11, the accuracy, sensitivity, determination, and *F*-criterion values of the classification made with DKSBS for the test data were calculated as 1. This means that the linguistic strong neurofuzzy classifier classifies all the test data correctly. Accuracy, sensitivity, determination, and F-measure values of the classification made with ANN for test data were also close to 1. This situation reveals that it is a method that can be used for test data, although it is more unsuccessful than the linguistic strong neurofuzzy classifier. All data clustered with *K*-means and *X*-means were used for training, so there are no accuracy, sensitivity, determination, and *F*-measure values calculated for the test data. The performance values of the study and the performance values of other studies were compared and found that different methods in different studies classified the same dataset. Still, no clustering process was found outside of this study. When the results of the studies are examined, it is seen that the success rate is above 90% in general, but there is also a study that is 100%. When the results obtained in this study are compared with the results obtained in other studies, it is seen that the classification success is higher when DKSBS and ANN classify the data than in studies classified with logistic regression, naive Bayes, fuzzy rule logistic regression combination, and j48 decision tree. The success rates of classification with fuzzy neural network architecture and classification with DKSBS within the scope of this study are the same. The accuracy in the data classified by the two methods is at the same rate, and this rate is 100%. This means that both methods correctly classify all samples. When the results of the clustering process carried out within the scope of this study are examined, it is concluded that the *K*-means method, one of the clustering methods, is more successful than the *X*-means method, and the success rate of both clustering methods is lower than the classification methods.

RETRACTED

## 4. Discussion

This study examined studies on OSB using techniques such as data mining and artificial intelligence. It is seen that many studies have achieved very successful results in this regard. In addition to this, the criticism that outdated datasets are used in the studies carried out in recent years with a scientific publications draws the attention [7]. When the details of the publication are examined, it is seen that technological developments are used by using current and successful methods. Still, it is emphasized that the data used in experimental studies are out of date. In the continuation of the study, outdated data, which is seen as a deficiency, were collected based on the last scale developed and shared after some operations were performed. The dataset includes 1100 samples, grouped as children, teenagers, and adults. This study used the subset for children containing 292 samples of the same dataset. Classification and clustering, which is one of the data mining methods [9], was applied to the dataset to estimate the output expressing the autistic status of the individual as a result of the inputs, which consisted of 20 inputs in total but were reduced to 19 after an attribute that was removed because it was the same in all samples. Before applying the classification and clustering processes, the missing data were first completed by looking at the frequency of the features on the dataset, which was completely converted to numeric values, and normalization processes were carried out. The dataset, which was prepared for the methods, was finally separated as 70% training and 30% test data. The data were classified as test and training data for the classification process, and the results were expressed with many parameters. The methods used for the classification process were ANN and DKSBS. Since the clustering methods are not pretutorial, the dataset is not separated as training and test, but it is clustered as all training data. *K*-means and *X*-means methods were used for clustering. Although the results obtained were expressed with many parameters, accuracy, sensitivity, determination, and *F*-measure were used to compare the common denominator in all methods. When the classification results are examined, it is seen that the success rate for the training dataset is 100% in two methods, namely, ANN and DKSBS [17].

RETRACTED

Therefore, the accuracy, sensitivity, determination, and *F*-measure values calculated for the training dataset of the two methods were calculated as 1. This means that both methods correctly classify all of the training data. When the results obtained for the test set are examined, it is seen that the success rates are different from each other. The success rate of the linguistic strong neurofuzzy classifier for the test data was the same as the success rate for the training data. Therefore, the accuracy, sensitivity, determination, and *F*-measure values calculated for the test set were calculated as 1. This means that all of the test data are correctly classified by DKSBS. The success rate of ANN for test data was 98.85%. Accuracy, sensitivity, determination, and *F*-measure values calculated for the test set were 0.989, 0.974, 1, and 0.987, respectively. These results mean that ANN classification misclassified only 1 of 87 samples in the test data and correctly classified the remaining 86 samples. Considering the success of classification methods [9], two methods are used.

## 5. Conclusion

The contributions of this study to the literature are as follows: when the studies conducted with the same dataset are examined first, it is seen that the classification processes are made by using methods such as logistic regression, Naive Bayes, fuzzy rule logistic regression combination, fuzzy neural network architecture, and j48 decision tree. Still, it is seen that the clustering process is performed with any method in the subset for children. Although no study has been found, a classification made with ANN and DKSBS has not been found. When we look at the results, it is seen that the classification methods are more successful than clustering methods in the data of ASD for children in terms of estimation accuracy. It is concluded that the DKSBS method can be one of the best methods that can be preferred, especially since it has a higher success rate than many methods in the literature by correctly classifying all the data. Therefore, it allows to try different methods for the dataset used in this study and allows classification with a method that has more successful results than many studies in the literature. In addition, the parameters used to evaluate the results obtained are given in more detail than many studies. This allows for a more detailed interpretation of the obtained results.

RETRACTED

### 5.1. Recommendations

In future studies, some analyses can be performed using different subsets of the dataset or using all subsets simultaneously. In future studies, studies that can be applied to more comprehensive datasets supported by different technologies such as decision support systems, expert systems, and image processing techniques can be carried out. New studies can be carried out jointly with the physician or physicians who are experts in the field to collect the data up-to-date. Then, concrete products that continue to learn and can be used in normal life can be revealed with the findings obtained.

## Figures and Tables

**Figure 1:** Performance of neural network.

**Figure 2:** ANN model with the highest success rate.

**Figure 3:** ROC curve plotted for the test data of the trained network.

**Figure 4:** Error matrix plotted for the test data of the trained network.

**Figure 5:** Educational performance of the linguistic strong neurofuzzy classifier.

**Figure 6:** Error matrix plotted for test data.

**Figure 7:** Error matrix plotted for the results obtained with the *K*-means algorithm.

**Figure 8:** Error matrix plotted for the results obtained with the *X*-means algorithm.

**Figure 9:** Performance values of the methods used.

**Figure 10:** Accuracy, sensitivity, determination, and *F*-measure values for the training datasets of the methods used.

**Figure 11:** Accuracy, sensitivity, specificity, and *F*-measure values for the test datasets of the methods used.

**Table 1:** Details of the attributes in the dataset.

	Attribute	Datatype	Description
1	Answer to question 1	Binary (0,1)	He usually notices small sounds when others cannot hear it.
2	Answer to question 2		It usually focuses on the whole picture rather than the small details.
3	Answer to question 3		In a social group, he can easily follow the conversation of several different people.
4	Answer to question 4		He finds it easy to commute between different activities.
5	Answer to question 5		He does not know how to continue the conversation with candidates.
6	Answer to question 6		He is good at social chat.
7	Answer to question 7		He has trouble deciphering the character's intentions or feelings when he reads a story.
8	Answer to question 8		While in preschool, she enjoys playing with other children.
9	Answer to question 9		You can easily tell what someone is thinking or feeling by looking at their face.
10	Answer to question 10		He has a hard time making new friends.
11	Age	Number	Information on how old the individual is in years.
12	Gender	String	Knowledge of whether an individual is male or female
13	Ethnicity	String	Information about the ethnic origin of the individual.
14	Being born with jaundice	Boolean (yes-no)	Information on whether an individual is born with jaundice.
15	Family members with PDD	Boolean (yes-no)	Information on whether the individual has any family members with PDD.
16	Country of residence	String	Information of the individual's country of residence.
17	Using the scanning application before	Boolean (yes-no)	Information whether the user has used a scanning application before.
18	Scoring result	Integer	The final score was obtained based on the scoring algorithm of the screening method used.
19	Who completes The test	String	The information of who performed the individual's test (parent, herself, caregiver, health personnel, clinician, etc.).
20	Autistic status (output)	Boolean (yes-no)	Knowledge of the individual's autistic status

RETRACTED

## Data Availability

The data underlying the results presented in the study are available within the manuscript.
